# Deep Transfer Learning Approaches in Performance Analysis of Brain Tumor Classification Using MRI Images

**DOI:** 10.1155/2022/3264367

**Published:** 2022-03-08

**Authors:** Chetana Srinivas, Nandini Prasad K. S., Mohammed Zakariah, Yousef Ajmi Alothaibi, Kamran Shaukat, B. Partibane, Halifa Awal

**Affiliations:** ^1^Department of ISE, Dr. Ambedkar Institute of Technology, Bengaluru 560056, India; ^2^Department of Computer Science, College of Computer and Information Sciences, King Saud University, P.O. Box 57168, Riyadh 21574, Saudi Arabia; ^3^Department of Computer Engineering, College of Computer and Information Sciences, King Saud University, P.O. Box 57168, Riyadh 21574, Saudi Arabia; ^4^School of Information and Physical Sciences, The University of Newcastle, Callaghan 2308, Australia; ^5^Department of ECE, SSN College of Engineering, Chennai, India; ^6^Department of Electrical and Electronics Engineering, Tamale Technical University,Tamale, Ghana

## Abstract

Brain tumor classification is a very important and the most prominent step for assessing life-threatening abnormal tissues and providing an efficient treatment in patient recovery. To identify pathological conditions in the brain, there exist various medical imaging technologies. Magnetic Resonance Imaging (MRI) is extensively used in medical imaging due to its excellent image quality and independence from ionizing radiations. The significance of deep learning, a subset of artificial intelligence in the area of medical diagnosis applications, has macadamized the path in rapid developments for brain tumor detection from MRI to higher prediction rate. For brain tumor analysis and classification, the convolution neural network (CNN) is the most extensive and widely used deep learning algorithm. In this work, we present a comparative performance analysis of transfer learning-based CNN-pretrained VGG-16, ResNet-50, and Inception-v3 models for automatic prediction of tumor cells in the brain. Pretrained models are demonstrated on the MRI brain tumor images dataset consisting of 233 images. Our paper aims to locate brain tumors with the utilization of the VGG-16 pretrained CNN model. The performance of our model will be evaluated on accuracy. As an outcome, we can estimate that the pretrained model VGG-16 determines highly adequate results with an increase in the accuracy rate of training and validation.

## 1. Introduction

Tumor is also termed as neoplasm produced by uncontrolled growth of anomalous cells [1]. A brain tumor (cancer) is a mass of abnormal tissues found in the central spinal canal or brain [2], wherein few cells grow and spread uncontrollably, ostensibly unregulated by the natural process that controls normal cells. Our brain is encapsulated by the skull, which is very intransigent. The tumor grows rigorously inside such a restricted space and hampers the natural functioning of the brain. The main cause of deadly cancerous cells in the brain can be associated with substantial conditions like the disproportionate inhale of inorganic chemicals or ancestral disorders. Brain tumors can take the form of benign (noncancerous) and malignant (cancerous). When benign, precarcinoma, or malignant tumors grow, the pressure inside the skull beneath increases causing several complications for humans. This will result in traumatic brain damage and can be life-threatening. Brain tumor detection at early stages is very important in increasing the human survival rate. Several techniques [1] were suggested for the prediction of tumors in the brain. Tumors in the brain organ are categorized into three types that are generally recognized as glioma, meningioma, and pituitary tumors [3]. Medical image technology in the e-healthcare domain plays a vital role in today's emerging field. Research of medical experts faces a lot of obstacles in identifying deadly brain tumor cells. Diagnosis of brain tumors at early stages has become a crucial task in medical science as it is ranked tenth in the leading diseases. Cancerous tumors of the brain occur at different locations and have varying dimensions and sizes.

Generally, to yield images of the human body's soft tissue, various techniques are used for medical image analysis. MRI images are one of them that are used by medical experts. It is a noninvasive technique used for accurate image data analysis of human brain tumors in determining the patient's condition [4]. It is highly applicable due to tissue contrast normalization and image quality resolution. The MRI images provide the genetics, physiology, chemistry, and biological information about abnormalities present in the brain [5]. Tumors are classified into several forms based on their origin and the nature of the cell. The primary vertebrate cerebrum tumors appear in the central hemispheres area, whereas secondary brain tumors locate their path from other human organs to the brain. The most common primary brain tumors are glioma, meningioma, and pituitary tumors in Figure 1.

Gliomas usually arise from the internal (gluey) cell of the brain. This cell, named the glial cell, helps in the proper functioning of brain neurons. World Health Organization (WHO), grade II-III glioma as non-glioblastoma and grade IV defined as glioblastoma [6]. There exist three forms of normal glial cells that produce deadly tumors [7]. Astrocytoma tumor will be produced by astrocyte cells (including glioblastomas), an oligodendrocyte will result from oligodendroglioma cells, and ependymoma occurs through ependymal cells. Tumors that include the combination of these distinctive glial cells are referred to as mixed glioma. Meningioma tumors arise from cerebral membranes that encapsulate the brain and spinal cord within the inner portion of the skull. Particularly, these passive growth tumors occur on the three membrane layers called meninges. Pituitary adenoma (tumors) arises abnormally in the pituitary gland region that exists inside the skull, between the brain and nasal passages. Meningioma and pituitary tumors are benign that do not escalate to other tissues, cells, and other parts of the human body. Glioma is a malignant tumor that spreads across the human body organs.

Image classification is an essential and extensive domain within the research area of deep learning and computer vision. Image classification refers to the process of assigning labels to an image into one of a number of predefined classes. The classification includes image data acquisition, image data preprocessing, image object detection, image segmentation, feature extraction, and image object classification. Image classification is the most significant and crucial task, especially in medical healthcare domains, including biomedical imaging, detecting, and diagnosing the disease accurately, which helps radiologists to improve diagnostic efficiency and provide a better path for surgical treatment.

### 1.1. Motivation

The brain tumour is a life-threatening neurological disorder that occurs due to the uncontrollable growth of abnormal cells in the human nervous system. Over the last twenty years, the incidence of brain tumours has been increasing in all ages. It has been predicted recently as the third most extensive cancer recognized majorly in adults and teenagers. Around the world, according to International Agency for Research on Cancer (IARC), proportionately more than 136000 populations are investigated for brain tumors per year, with more than 87000 loss of survival rate in 2017 [8]. Medical experts put inconsistent effort to conquer the complications of brain tumors; According to the World Health Organization (WHO) statistics, it is estimated that 251,329 people die from cancerous brain disease approximately every year. Therefore, accurate brain tumor diagnosis is an essential task for patient survival and providing effective medical treatment. Recently, many researchers proposed various multidisciplinary models, including medical science knowledge, mathematics, and computer science, to understand the disease and identify more adequate surgical methods. Various image modalities are referred for brain images data analysis, such as Magnetic Resonance Imaging (MRI), Single Photon Emission Computer Tomography (SPECT), BIOPSY scan, and computer tomography (CT). The most common imaging techniques are MRI and CT undertaken for brain scans to predict the existence of brain tumors and to identify their position for preferred professional treatment benefits. The proper treatment options depend on the brain tumor's location, size, shape, category, and grade. Medical treatment options also depend on whether or not the tumor is spreading and affecting the other organs of the body or within the part of the central nervous system (CNS).

### 1.2. Importance of MRI Biomedical Image Processing

Therefore, an MRI scan is considered the most efficient tool compared with other image modularities. A well-experienced radiologist can investigate the brain MRI scan and decide on treatment options based on the type of tumor [9].

MRI [10] is one of the essential imaging techniques used precisely in brain tumor detection. Brain tumor is one of the most deadly diseases occurring in the central nervous system of the human body. MRI medical imaging technique uses a very powerful magnet, magnetic field gradients, and computer-generated radio waves to scan and display internal organ images within the human body. MRI scan plays a vital role for healthcare professionals in examining brain tumors to provide better patient treatment. MRI is an analytical development in the medical field that produces high-resolution images to detect and diagnose tumor existence in the human brain organ. MRIs create more detailed high-quality images than CT scans. It uses magnetic radio waves to scan the organ within the body.

Therefore, an MRI scan is considered the most efficient tool compared with other image modularities. A well-experienced radiologist can investigate the brain MRI scan and decide on treatment options based on the type of tumor. Investigation of the MRI medical image by the radiologist is a time-consuming process, and the efficiency in decision-making confides their expertise in the medical field. Therefore, a computerized brain tumor classification process helps radiologists in their investigation and reduces their interferences extremely.

### 1.3. Why Deep Learning Methods?

Machine learning techniques are the first automation classification methods in the image classification process for detecting deadly tumor diseases. Due to the need for preprocessing of image data and extraction of distinct features in MRI images, they take a long time to classify the tumor. The main disadvantage of machine learning methods is that classification process accuracy mainly depends on handcrafted features identified by feature extraction methods. Acquisition of data based on different algorithms is one of the significant challenges. The acquired data can be highly error-prone, as the data required for training the model must be clean, structured, and accurate. Also, the selection of machine learning algorithms for a particular problem is based on data collection; additionally, machine learning algorithms take more computational time to process a huge amount of data. In spite of machine learning methods limitations, some researchers proposed methods and achieved classification accuracy rates of 78% and 86% based on textual or statistical feature extraction methods.

Artificial intelligence and advanced deep learning models based on transfer learning and artificial neural networks achieved a higher classification accuracy rate in self-learning the image features to classify MRI images without the need for feature extraction methods suggested by [11, 12]. Transfer learning is a predefined approach in deep learning or machine learning used to speed up deep learning training. The pretrained models can be used to solve complex problems with preexisting knowledge. These models provide rapid advancement in the medical field to assist medical experts in investigating and diagnosing cancerous tumors at early stages. To solve complex issues in real-time functionalities and also in the processing of image feature extraction, classification, localization, and detection, CNN with a transfer learning approach is an important image processing technique worn for analysis of medical data imaging among various deep learning methods [13].

## 2. Literature Survey

In recent years, an enormous number of approaches to brain tumor classification on MRI brain images have been proposed based on deep transfer learning models. CNN was realized as the first real-world application in 1998 to observe handwritten digits [10]. Premamayudu Bulla et al. [14] developed a hybrid model based on CNN for classifying the tumor type in the brain. Hassan Ali Khan et al. [7] proposed an automated brain tumor detection mechanism applying CNN with transfer learning models on the MRI brain image dataset. The effect of MRI image data preprocessing steps analyzed by authors [15] improves the classification accuracy in predicting brain tumor disease. Researchers [16] focused on developing a new CNN-based model to classify the three forms of tumors that existed in brain MRI images. Toktam Hatami et al. [15] investigated presenting a CNN pretrained model with image segmentation techniques. Venkatesan Rajinikanth et al. [17] suggested a VGG-16 pretrained CNN model for the classification of multigrade brain tumors. ImageNet Large-Scale Visual Recognition Challenge (ILSVRC), a visual database project, was launched by ImageNet in 2010. This challenge provides a platform for many researchers to analyze the performance of proposed methodologies developed on the given image dataset and obtain a higher classification accuracy rate. Muhammed Talo et al. [4] proposed CNN architecture AlexNet to achieve good results on various tasks based on visual recognition. The major obstacle in the development of the deep neural network in the medical field was the lack of labeled image datasets. This is overcome by applying a data augmentation approach to increase the volume of data from available labeled image datasets for a better accuracy rate. CNN-based transfer learning models accomplished excellent performance in the medical healthcare field due to the capability of self-feature learning without any human expert; weight sharing provides an adequate impenetrable network to perform automatic prediction or detection of disease through MRI brain images. Since 2014, according to the statistics analysis gathered from researchers, the number of CNN-based publications in general in the medical image appliances and specifically for brain tumor disease has been rapidly expanded. In today's scenario, brain MRI image datasets are publicly accessible for medical scientists [18]. This assisted medical investigators in proposing further new automation classification models for prediction or detection purpose used for medical applications. H. Mohsen et al. [19] developed computer-aided diagnosis (CAD) system for automatic detection of brain tumors in brain MRI images. The proposed model utilizes sequential minimal optimization (SMO) algorithm for training Support Vector Machine (SVM) to classify glioblastoma, sarcoma or metastatic bronchogenic carcinoma malignant tumors. S. T. Kebir et al. [20] designed an automatic and a supervised MRI Brain abnormalities detection methodology. The proposed method undergoes with three parts such as construction of CNN deep learning network, segmentation using K-Means algorithm and classification of normal or abnormal brain cases.

The main purpose of this paper is to adopt a deep transfer learning approach with CNN pretrained models such as VGG-16, Inception-v3, and ResNet-50 to perform brain tumor disease detection. Based on training time and epoch number, this work presents the overall classification accuracy rate of three pretrained architectures [21]. To minimize the computation time in prediction of disease, we explore the significance of epoch numbers. Lastly, this work explains the comparative performance analysis of deep transfer learning-based pretrained models on a classification of brain tumor disease through MRI.

The drawback of the previous work relies on detection of tumors from either glioma, meningioma, or pituitary brain tumor types in predicting the tumor [22]. The limitations of the existing approaches were not performed without specifying the tumor type and its grade level. The CNN with pretrained models is implemented using the Keras and modularities TensorFlow due to its high performance in detecting cancerous tumor cells.

## 3. Methodology

### 3.1. Dataset Collection and Preprocessing

The dataset acquired in this study is a collection of images of brain MRI scans. There exist around 256 raw MRI images of different dimensions (width *∗* height), usually measured in terms of pixel values. The sample MRI brain images are gathered from the Kaggle dataset. The collected images are in Joint Photographic Experts Group (JPEG) format [23]. The image database is categorized into two segments, Yes and No, based on the existence of the tumor in an MRI brain image. Benign tumors are around 158 brain MRI images and the remaining 98 brain MRI images are malignant tumors. Generally, in our work, we split our dataset into three segments required for training, testing, and validation. The sample MRI brain image dataset is shown in Figure 2.

The steps involved to preprocess Kaggle's brain image dataset [24] before applying CNN pretrained models are as follows:

(1) Import the packages needed.
(2) Import the two data folders with “Yes” and “No.”
(3) Read the images and transform them as labeled images (Tumor = Yes and No Tumor = No).
(4) Store labeled MRI images in the data frames.
(5) Resize the images with the dimension of 256 × 256.
(6) Normalize the images by image cropping by using the mathematical equation
  (1) $$\begin{array}{c} i=\frac{i\;-\mu_{i}}{\sigma_{i}}. \end{array}$$

The MRI images available in the dataset were preprocessed in the following manner shown in Figure 3.

Intensity normalization is a major step in brain MRI analysis. During image data acquisition, a variety of scanners would be used for scanning the images at different time-period, which may result in large variations in pixel intensity [25, 26]. Therefore, overall pixel values in multiple images are normalized into the same statistical distribution required for better analysis of MRI images.

Due to MRI machinery limitations, anomalies could be found in MRI brain images. The abnormalities such as poor quality image resolution, distortion, inhomogeneity, misinterpretation, and motion heterogeneity are produced by limitations in MRI image processing. These inaccurate analyses of scanned images could result in false positives while investigating the brain MRI image. This poor diagnosis further affects patient treatment options. The CNN-pretrained models require the brain MRI to be resized with a 224 × 224 × 3 dimension [11], so the dataset MRI images are reformatted to a specific dimension.

Firstly, the input MRI images are cropped to include the brain portion only from MRI brain images with open-source computer vision (CV). Many of the researchers developed various computer-aided diagnosis (CAD) models on publicly available small datasets [27]. But, we know that state-of-the-art deep transfer learning models require a large volume of data to obtain a better optimized classification accuracy. Therefore, a huge voluminous dataset is required to train the CNN model to minimize the probability of overfitting problems. In order to overcome limited datasets, this study utilized a transfer learning preprocessing technique called data augmentation. Among several techniques, namely, scaling, cropping, resizing, flipping, rotation, and perspective transformation, a specific technique is applied based on the requirement.

It is a method used for generating artificial image data for training from the original dataset [28]. Artificial data augmentation is useful to increase the performance of the proposed diagnosis model by producing new and distinct data examples required to train the model.

The experimental results signify that the deep learning-based CAD model trained with artificial augmented data works better and gives accurate results to train the model as compared with the real image dataset.  Figure 4 shows the augmented MRI brain image dataset [29]. The data augmentation methods, namely, affine image transformation approach, and pixel-level image transformation methods are applied to produce the new training examples to train the model.

### 3.2. Convolution Neural Network (CNN)

Advanced artificial intelligence models based on a deep transfer learning approach are highly efficient for medical disease prediction problems based on image classification [30]. Deep neural networks based on CNN or ConvNets are networks that include some mathematical or linear operations called “convolution.” A convolution neural network (CNN) is an architecture of several levels observed like multiple hidden layers, pooling layers, and output layers or fully connected (FC) layers. These hidden layers are named a sequence of convolution layers with filters (kernels) that performs image classification operation in predicting patients' diseases [31]. The pooling layer reduces consecutively spatial size representation and decreases hyperparameters. Expensive computation in ConvNet is reduced by the pooling layer. Thus, the overfitting problem in ConvNet is resolved. CNN is one of the categories of artificial neural networks that do not require handcrafted feature extraction in advance to classify the MRI brain images. Finally, the network also consists of ReLU-activated segments of 3096, 3096, and 1200, respectively. The mathematical formula for expressing ReLU is as follows:

(2) $$\begin{array}{c} f\left(y\right)=\max\left(0,y\right). \end{array}$$

The ReLU plays a significant role in improving the neural networks by speeding up the training phase. Also, the computational steps of ReLU are simple and easy with negative values set to zero and having no exponentials, division, or multiplication operations on the training dataset.

The input MRI images are resized into 256 × 256 to overcome the overfitting problem. CNN models involve a series of layers with filters to perform the task of dimension reduction and feature extraction. Therefore, CNNs are termed as “feature extractor” that can extract significant features, analyze them on their own, and classify features efficiently [32]. To generate the result, the FC layer is used with the required set of classes to perform a nonlinear transformation on the extracted features, further operating as an image classifier to analyze and classify MRI brain images. The general CNN structure is shown in Figure 5.

The feature vectors are extracted from fully connected layers of CNN and further passed as an input to 1000 units of softmax layer for classification.

Mathematically, the equation for the softmax activation function is as follows:

(3) $$\begin{array}{c} \sigma {\left(z\right)}_{i}=\frac{e^{z_{i}}}{\sum_{j=1}^{K}e^{z_{j}}}. \end{array}$$

Here, “*z*” is the softmax function input vector consisting of “*n*” features of “*n*” target values (outcomes), “*zi*” is the *i*th item of the input vector which can take the values either positive “+” or negative “−,” “*e*^*zj*^” is the standard exponential function implied on *xi*, and “Σ *e*^*z*^_*j*_” is a normalization term to obtain the valid probability distribution.

The implementation of our proposed model is done in Python programming language and executed in Anaconda Jupiter Notebook, Google Colab. The method is trained with 120 epochs with the training, testing, and validation dataset.

### 3.3. Transfer Learning Approach

Advanced deep learning models [7] based on transfer learning demands huge volumes of data for training and executing optimally state-of-the-art high processing resources and sufficient time to train the model. Transfer learning finds a solution to another task by utilizing knowledge gained from previously learned task [27, 33]. It is an approach of utilizing pretrained CNN models based on parameter fine-tuning for computing identical tasks. In deep learning, the transfer learning approach is used with already available pretrained models trained on a huge voluminous dataset like ImageNet for image classification instead of developing the CNN detection model [34] from scratch to classify the image.

The healthcare data acquisition is usually a small sample size since it is very difficult to extract. Further, it is processed with the pretrained model ImageNet, mainly used for natural images. As there are a lot of differences between natural images and MRI images, we need to fine-tune our model with transfer learning methods with CNN-based pretrained hyperparameter models [5].

This approach is used when the dataset size is small for training and extensively adopted for computer vision-based problems. Transfer learning generally works on acquiring the ImageNet dataset as an input. The convolution layers freeze, and weights with a particular dataset are transferred to other CNN models and then generate the final image classification as an output [22]. Therefore, in a nutshell, it is called an improved learning model for new tasks by transforming knowledge gained from existing tasks. The general working principle of transfer learning is as shown in Figure 6.

### 3.4. CNN-Based Deep Learning Model

The proposed work incorporates the process of automatic detection and diagnosis model for the prediction of brain tumors in MRI images. The steps involved in the proposed approach are as illustrated in Figure 7. The first step incorporates the acquisition of data in the form of MRI brain images from the Kaggle dataset [35]. Each individual image is further gone with various preprocessing techniques, namely, resizing, cropping, and pixel-level data augmentation. Later, preprocessed images were processed with the training and testing phase through CNN pretrained models for predicting the disease in the brain.

Our proposed research study makes use of CNN with pretrained architectures to train the model to predict the disease. The CNN deep learning brain tumor-based classification is split into two divisional phases, training phase and testing phase. The performance evaluation of the model is carried out in two phases based on the splitting of the acquired dataset as training and testing phases. The MRI brain images are categorized as tumorous and nontumorous MRI images. In our study, we considered three types of brain tumors like glioma, meningioma, and pituitary brain tumors.

In this proposed model, a pretrained CNN architecture is employed for the classification that uses many labeled images for training the model obtained from large-scale datasets like the ImageNet and Kaggle.

For our research work, three pretrained CNN architectures like VGG-16, Inception-v3, and ReseNet50 are used for classification purposes. The block diagram in Figure 8 represents the methods adopted in our proposed approach.

The dense layer plays a significant role in classifying the brain MRI image based on outputs from the convolution layers [29]. It feeds outputs from the previous layer to all its neurons; each individual neuron provides one output to the next layer.

### 3.5. CNN-Based Pretrained Models for Image Classification

CNN-pretrained architectures applied in this work are VGG-16, Inception-v3, and ResNet50 to classify MRI brain tumor problems using a transfer learning approach.

#### 3.5.1. VGG-16 CNN Model

In our experimentation, we applied the VGG-16-pretrained CNN model. Because of the small image dataset and to avoid overfitting problems, our model is fine-tuned by freezing some of the convolution (Conv) layers. VGG-16 is a CNN model with sixteen convolution layers developed in 2014 by researchers [15]. The model accepts brain MRI images as an input with a dimension of 224 × 224 × 3. It incorporates Conv layers with kernels (filters) of fixed 3 × 3 filter size and 5 max-pooling layers of dimension 2 × 2 in size within the network [36]. It also includes extensively ReLU activation functions and 2 fully connected layers with a softmax output layer. VGG-16 model is a broad network that contains approximately 138 million hyperparameters. It stacks multiple convolutional layers to construct deep neural networks that improve the ability to learn invisible handcrafted features. The hyperparameters are essential as they control the overall behavior of the model. Its aim is to minimize the predefined loss function and to obtain better results for a specific dataset. The hyperparameters to tune are the neuron and epoch counts, softmax activation function, learning rate, and optimizer. The number of convolution layers is the second step of the hyperparameter to undergo tuning.

Thus, with an increase in ConvNet depth, the capacity to learn hidden features increases with a lower cost. In Figure 9, the VGG-16 ConvNet architecture is shown.

#### 3.5.2. Inception-v3 CNN Model

Inception CNN network named GoogleNet was introduced and developed by Google Brain Team in 2014, trained on ImageNet database. Inception was a pretrained network of 22 layers including 5M parameters with a kernel (filter) dimension of 1 × 1, 3 × 3, and 5 × 5 to capture handcrafted features at different scales, including the max-pooling layer. The reason to use filters with 1 × 1 kernels is to preserve computation time with less impact on network performance. Later in 2015, Google extended up the Inception network to Inception-v3 [5], in which Conv layers are rescaled to decrease with hyperparameters. Inception-v3 is a 48-layer deep neural network, which classifies MRI brain images into thousand image classes and also avoids overfitting problems.

The model has the self-learning capability to extract various images' handcrafted features and analyze them for brain image classification. The Inception-v3 network [3] requires an input image of dimension 299 × 299. Inception-v3 utilizes batch normalization, RMSprop, and image distortion for better performance in computer vision problems.  Figure 10 represents the basic architecture of the Inception-v3 model.

#### 3.5.3. ResNet50 CNN Model

ResNet50 comprises a 50-layer Residual Network with 26M parameters introduced by Kaiming He et al. at Microsoft Research in 2015 [12] for image recognition and classification. In Residual Network, the term residual is termed as feature subtraction. Instead of learning features, we learn from those features that are subtracted and learned from the layer's input. When compared with conventional deep CNN, ResNet50 is comparatively simpler to train. The pretrained model is trained on the ImageNet database [1]. These networks also overcome degrading image classification accuracy problems. It includes skip connections in addition to enormous batch normalization. These skip connectivities are specified as gated recurrent units or gated units. ResNet50 network establishes a direct connection between *n*th layer input to some (*n* + *x*)th layer, which propagates additional layers to be stacked in order to construct a deep neural network. This Residual Network has a lower time complexity when compared with VGG16 or VGG19 models. In our experiment, we adopted a pretrained ResNet50 model and calibrated it to suit the input image dataset. The pretrained architecture of ResNet50 is shown in Figure 11.

### 3.6. Performance Evaluation Metrics

Image classification plays a prominent role in healthcare applications to detect and predict deadly cancerous tumors in human body organs. Most popular image classification models are, namely, convolution neural network, Recurrent Neural Network, Support Vector Machine, Random Forest, Logistic Regression, and many advanced deep learning models based on transfer learning methods. The performance of various classifiers for predicting disease can be evaluated by several metrics such as accuracy, precision, recall, and F1-score. The sensitivity and specificity are associated with classification accuracy, which uses the terms true negative (TN), true positive (TP), false negative (FN), and false positive (FP). In the field of deep learning, one of the important techniques for summarizing the performance of image classification is the confusion matrix. It is also known as an error matrix, a tabular design that allows performance visualization of the predictions and truth labels in the classification model. In predictive analysis, each row of a confusion matrix represents the instances in an actual class, and each column represents an instance in the predicted class and vice versa. The diagonal elements of the error matrix represent correct classification predictions, and nondiagonal elements represent the incorrect image classification prediction. The output of the confusion matrix is in terms of true positive (*tp*), true negative (*tn*), false negative (*fn*), and false positive (*fp*). The above terminologies are used to calculate accuracy, precision, recall, F1-score, sensitivity, and specificity to estimate the performance of classification models, as shown in Table 1 [2].

Most model performance measures are based on the model's prediction with the dataset values. They are computed for the training dataset, a data used for learning the model. The CNN classifier leads to a confusion matrix if classification is of double class issue shown in Table 2.

### 3.7. Performance Result Analysis and Discussion

This segment discusses the performance evaluation of pretrained CNN architectures in findings of the MRI brain tumor image classification. The accuracy, precision, recall, and F1-score along with the training time of the model are shown in Table 3. The pretrained CNN classification architectures VGG-16, Inception-v3, and ResNet50 are implemented on the brain MRI dataset containing 253 brain MRI images, of which 154 images are of the affected cancerous cells.

The VGG-16 has a total of 138 million hyperparameters, all the convolution kernels are of the size 3 *∗* 3, and max-pool kernels are of the size 2 *∗* 2. This reduces the number of trainable datasets by 44.9% out of 100%. The reduced trainable data means a faster learning rate and overfitting problems. The Inception-v3 consists of various Inception modules; each module that exhibits the four operations in parallel helps in depth reduction of convolution layers. ResNet50, a pretrained CNN model, helps to train the model easily with an enormous number of convolution layers without increasing the training error rate.

The original image size was in various dimensions, on an average larger than 1000 × 1000 pixels. It is then resized to a dimension of 160 × 160 pixels and forwarded as an input image to a VGG-16 classifier as in Figure 12. The performance of classifiers is measured in terms of metrics like accuracy, loss, validation_loss, and validation_accuaracy. The experiments were performed on a Kaggle kernel, a cloud-based processing platform for artificial intelligence and data science projects using GPU virtual machines and RAM that empowers collective and reproductive analysis. The following represents graphs of each test predictive analysis along with 74 epochs, where the *x*-axis indicates an epoch and the *y*-axis represents accuracy and loss levels. The performance evaluation of the pretrained models is visualized in tabular form for the classification of the MRI image. Each row represents predicted classification target values, while columns represent the true classes from the training dataset.

#### 3.7.1. VGG-16 CNN Architecture

The predicted accuracy with VGG-16 along with accuracy loss, validation loss, and validation accuracy is as shown in Figures 13 and 14, respectively.

In VGG-16, training and validation accuracy represents a positive pattern and tends to rise up to 0.96% at each epoch interval. Similarly, there is a stable increase in validation loss with 0.95% at each epoch interval, and validation loss tends to decrease till the final epoch. The training accuracy leads to how the proposed model is able to classify the two images during training on the trained dataset, while validation accuracy deals with classifying the images with the validation dataset. Meanwhile, the training loss implies how well the model is fitting the training dataset, while the validation loss indicates how well the model fits the newly acquired MRI image data. The performance of prediction made by the VGG-16 classification model is shown in the confusion matrix as illustrated in Figure 15, where each row indicates the actual class and each column indicates the prediction class. This is a sample to identify how well the model is predicted from the testing data, classifying 17 out of 19 nontumorous images and 27 out of 31 tumorous images.

#### 3.7.2. Inception-v3 CNN Architecture

In Inception-v3, training accuracy shows that the graph tends to rise while validation accuracy is unstable. The highest increase in validation accuracy occurs after the 8th epoch reaching 0.86% from the 4th epoch of 0.78%; validation loss shows a graph with unstable results, while training accuracy tends to rise with stable results until the last epoch as in Figures 16 and 17. The confusion matrix result of the Inception-v3 model predicting from testing data and classifying 18 images out of 19 images as false positive is shown in Figure 18.

#### 3.7.3. ResNet50 CNN Architecture

In the ResNet50 test, the resulting training accuracy is increasingly higher and stable from the 2nd epoch to the last epoch, reaching accuracy above 0.95%, while the validation accuracy that is unstable tends to rise at the 5th epoch and poor performance conditions after the 8th epoch at 0.78% cannot predict the new class of data accurately illustrated in Figures 19 and 20, respectively. The performance results of the ResNet50 model are expressed in a confusion matrix predicting tumors from the testing data and classifying 11 MRI brain images out of 31 images as a false negative, which is the drawback of this model as in Figure 21.

## 4. Conclusion

This research presents a comparison of deep pretrained convolution neural networks based on transfer learning architectures, which naturally classify brain MRI images as benign and malignant tumors. The image classification process is performed using transfer learning pretrained CNN architectures, namely, VGG16, Inception-v3, and ResNet50, which acts as a classifier in prediction analysis in brain tumor detection. Data preprocessing, data augmentation methods, and hypothesized hyperparameter integral tuning are added in each testing step. Pretrained CNN architecture is said to give better performance results if, for each epoch, training accuracy and validation accuracy increase. The architecture is predicted to undergo overfitting problems, specifically when validation accuracy decreases while training accuracy increases. The model suffers an issue of overfitting when it cannot make proper predictions for a new dataset and is limited to focusing on particular training data. With the evaluation performance of each architecture, it shows that all architectures gain training accuracy of more than 0.9000%, with the highest validation accuracy reaching 0.8826%. From the performance analysis of various pretrained CNN models, namely, VGG-16, Inception-v3, and ResNet50, we conclude that we found that VGG-16 gives better accuracy on the trained and tested dataset. And also validation accuracy is much nearer to the accuracy with less loss and validation loss.

The proposed study focused on only three pretrained models, namely, VGG-16, Inception-v3, and ResNet50, for image classification based on various tumor types. The research work can further be extended for classification with others like VGG-19, MobileNet, and EfficientNet-pretrained CNN-based models in the predictive analysis of brain tumors.

## Figures and Tables

**Figure 1:** Typical brain tumor types.

**Figure 2:** Sample dataset of brain MRI images.

**Figure 3:** Steps involved in MRI image dataset preprocessing.

**Figure 4:** Augmented brain MRI image dataset.

**Figure 5:** General CNN structure.

**Figure 6:** Transfer learning model.

**Figure 7:** The flow diagram of the proposed approach.

**Figure 8:** A block diagram representation of the methods used for this proposed study.

**Figure 9:** VGG-16 model architecture.

**Figure 10:** Inception-v3 model architecture.

**Figure 11:** ResNet50 model architecture.

**Figure 12:** VGG-16 classification process loaded with MRI image data [22].

**Figure 13:** Training and validation loss curve of VGG-16.

**Figure 14:** Training and validation accuracy curve of VGG-16.

**Figure 15:** Confusion matrix results of the VGG-16 model.

**Figure 16:** Confusion matrix results of the Inception-v3 model.

**Figure 17:** Training and validation loss curve of the Inception-v3 model.

**Figure 18:** Training and validation accuracy curve of the Inception-v3 model.

**Figure 19:** Training and validation loss curve of the ResNet50 model.

**Figure 20:** Training and validation accuracy of the ResNet50 model.

**Figure 21:** Confusion matrix results of the ResNet50 model.

**Table 1:** Performance evaluation metrics for classification models [2].

Metrics	Formula	Evaluation focus
Accuracy (acc)	(tp+tn)/tp+fp+tn+fn	In general, the accuracy metric measures the ratio of correct predictions over the total number of instances evaluated.
Error rate (err)	(fp+fn)/tp+fp+tn+fn	Misclassification error measures the ratio of incorrect predictions over the total number of instances evaluated.
Sensitivity (sn)	tp/(tp+fn)	This metric is used to measure the fraction of positive patterns that are correctly classified.
Specificity (sp)	tn/(tn+fp)	This metric is used to measure the fraction of negative patterns that are correctly classified.
Precision (p)	tp/(tp+fp)	Precision is used to measure the positive patterns that are correctly predicted from the total predicted patterns in a positive class.
Recall (r)	tp/(tp+tn)	Recall is used to measure the fraction of positive patterns that are correctly classified.

**Table 2:** Confusion matrix [37].

	Positive prediction	Negative prediction
Actual positive	TP	FN
Actual negative	FP	TN

**Table 3:** Performance evaluation metrics.

Model	Accuracy	Precision	Recall	F1-score	Time (sec)
VGG-16	0.96	0.94	1.0	0.98	3055
Inception-v3	0.78	0.75	0.70	0.73	6512
ResNet50	0.95	0.92	0.89	0.94	8076

## Data Availability

The dataset used in our research work is from the Kaggle dataset, which is openly available for experimentation.
